# Influences of viewing angle, product position, and consumers’ physical characteristics on their Kansei images

**DOI:** 10.1371/journal.pone.0276421

**Published:** 2022-10-26

**Authors:** Chii-Zen Yu, Fong-Gong Wu

**Affiliations:** 1 Department of Animation and Game Design, Toko University, Chiayi, Taiwan; 2 Department of Industrial Design, National Cheng Kung University, Tainan, Taiwan; Hiroshima International University: Hiroshima Kokusai Daigaku, JAPAN

## Abstract

Changes in consumer behavior in recent years have led to a steady increase in the number of online shoppers. The viewing angle of a product and its position on a webpage can affect consumers’ Kansei images and purchase intentions. This study aimed to determine the influences of product viewing angle and position on a webpage on consumers’ Kansei images; the influences of consumers’ physical characteristics (i.e., sex, dominant hand, and dominant eye) on their Kansei images were also explored. An experiment was designed to evaluate the influences of viewing angle and position on consumers’ Kansei images. A product’s viewing angle and position on the webpage in question served as independent variables, and the participants’ Kansei images served as the dependent variable. Seven representative viewing angles were selected. A predetermined product was placed in nine positions in a 3×3 grid on a webpage. A total of 63 combinations were obtained, and an experiment and interview were designed to investigate the participants’ Kansei images for all 63. The following conclusions were drawn: 1. Viewing angle affected the participants’ Kansei images; 2. the position of the product on the webpage affected the participants’ Kansei images; and 3. some physical characteristics affected the participants’ Kansei images. In summary, online marketing platforms could document shoppers’ physical characteristics to provide them with personalized product displays in order to cater to their Kansei images preferences. These research findings could be applied to online shopping platforms, which could attract more diverse groups of clients by adjusting product display angles and product positions on webpages based on consumers’ physical characteristics and preferences.

## Introduction

This study investigated the influences of a product’s viewing angle and position on a webpage on consumers’ Kansei images. A literature review on consumers’ physical characteristics, Kansei engineering, and viewing angles and cognition was conducted. Regarding the dominant hand, the proportion of right-handed people notably surpassed that of left-handed people. Approximately 90% of the analyzed people were right-handed; only 10% were left-handed [1]. The field of view (FOV) differed by color shade as well as by sex. In general, men’s FOV was smaller than women’s, and the right-eye FOV was smaller than the left-eye FOV. Parsons claimed that the dominant hand and dominant eye affect sesorimotor coordination [2]. Lund found that when people used both their dominant hand and dominant eye, they attained optimal scores on the target hitting test [3]. Freeman and Chapman adopted a pursuit task to study hand–eye coordination and obtained results consistent with those of Lund [4].

Most research on physiological characteristics is in the fields of physiology, medicine, or sports [5–10]. Mohr found that right-handed people prefer to turn left, and left-handed people prefer to turn right. This difference in steering behavior may be due to a dopamine asymmetry between the cerebral hemispheres [5]. Gorynia studied the relationship between hand–eye preference and speech ability in healthy adult men and women with right-handedness [6]. Fagard found no relationship between dominant hand and dominant eye and reading ability [7]. Erhan and Gerek investigated the relationships among the dominant hand, dominant eye, dominant ear, and exercise rhythm of athletes [8]. Witkowski et al. studied the cognitive steps taken by customers when they booked a room online and the effects of website aesthetics on their booking intention [9]. Foutch and Bassi proved the relationship between the dominant eye and monocular vision threshold [10]. These results demonstrate that physiological characteristics have a certain degree of influence on the human body’s abilities and cognition.

Hardyck and Petrinovich compiled ten relevant studies on the dominant hand and dominant eye and found six studies indicating that the dominant eye for most right-handed people is the right eye; their other four studies did not identify a significant relationship between the dominant hand and dominant eye [11]. Adams recruited baseball players as participants to study the influence of the dominant eye on baseball hitting [12]. Regarding the relationship between viewing angle and cognition, Eerland et al. [13] designed two experiments involving the participants standing on a Wii balance board; the board was tilted 2° alternately to the left and right, and the participants did not perceive the tilt. The participants were then asked to estimate answers to test questions. Compared with the answers they gave when standing upright, the participants tended to underestimate values when tilted to the left and overestimate values when tilted to the right. Wu et al. [14] proposed that the optimal viewing angle of a Nokia 8250 was when the cellphone was rotated to the right and tilted upwards. Most of the participants expressed a liking for the following sets of angles: (X = 30°, Y = 30°), (X = 30°, Y = 15°), and (X = 30°, Y = 45°). Chaung [15] designed an experiment to identify the observation thresholds of various components’ feature shapes to serve as a basis for product image presentation. Such thresholds provide a reference range for product image displays for shopping channels when consumers cannot access physical products. The researcher concluded that the optimal viewing angle was an x-axis tilt of −45°~45° and y-axis tilt of −15°~15°. Chang and Chen [16] conducted a questionnaire survey on the viewing angles and Kansei images of cars displayed on webpages to explore the viewing angles that best represent cars’ sense of speed, stylishness, and steadfastness. The results can serve as a reference for interface design personnel in designing viewing angles for display cars.

In 1986, Yamamoto proposed Kansei engineering for designing the exterior of automobiles. Japanese scholar Nagamachi named the "emotional engineering" previously proposed as " Kansei engineering" and studied it in depth. Kansei is a psychological feeling that consumers produce about products. The purpose of Kansei engineering is to design new products according to consumers ‘feelings and needs, and to “transform” or “correspond” people’s feelings to the design elements when designing products. The sensibility has to be presented qualitatively, and it is known from the exploration which design decisions are in line with people’s sensibilities. Kansei engineering has been applied in different design industry fields, such as bicycles, automobiles, construction, magazines, cosmetics and other related product development.

Kansei engineering builds a series of adjectives from the five senses (vision, hearing, smell, taste, touch) to describe and help designers master the customer’s perceptual perception and psychological needs. Systematically embed user needs into the prototype design. Since vision plays an extremely important source of information in human life, the images studied by psychology are usually mainly based on visual images, as well as design-related academic research.

Studies have applied Kansei engineering to the design of beverage bottle, office chair, automobiles and electrical appliances [17–19]. Jindo and Hirasago applied Kansei engineering and quantification theory type I to car interior design to determine the relationships between Kansei images and the styles of car dashboards, speed pointers, and scales, in order to determine the safest combination [20]. Horiguchi and Suetomi applied Kansei engineering to the design of car-driving systems using a driving simulator [21]. Lai et al. discussed the association between imported and domestically manufactured cars with respect to style and affective elements; the researchers used Kansei engineering to explore correspondence between a car’s viewing angle and its style and affective elements [22].

Kansei engineering is used to support construction machinery design as a scientific method of incorporating human sensibilities into applied design [23]. Guo et al. present the integration of KE models and Genetic Algorithm is employed to search for a mini digital camera design scheme [24].

The aforementioned studies have all discussed the relationship between individuals and product characteristics or affective elements. The present study referred to these studies for the selection of product viewing angles to investigate the relationships of Kansei images with viewing angle and position and discuss the influence of viewers’ physical characteristics on Kansei images.

## Methods

The Kansei engineering procedure involves setting the theme, collecting Kansei vocabularies, conducting a survey, analyzing the results, and determining the design concept.

1. Setting the theme
  The orientation of the design is chosen, and the target consumers or markets are specified. Kansei engineering attempts to precisely quantify consumers’ intangible feelings into the orientation of product design on the bases of their experiences and feelings.
2. Collecting Kansei vocabularies
  A preliminary design concept is formed once the theme is set. A semantic space is built based on the feeling that a product evokes in consumers. Kansei vocabularies most relevant to the product to be designed are selected so that consumers experience corresponding feelings and feedback. The collection of Kansei vocabularies for this study refers to those mentioned in the literature with the design of wine glasses.
3. Conducting a survey
  As previously mentioned, Kansei engineering is mainly consumer-oriented. Therefore, an instrument allowing for statistical analysis of customer experience and feedback is required, and the data can serve as a reference for product design.
4. Analyzing the results and determining the design concept
  After analysis of consumer experience and feedback, a preliminary design concept is obtained.

An experiment was designed to discuss the influence of a product’s viewing angle and position on a webpage on consumers’ Kansei images. Images with seven representative angles were selected (Figs 1–7) and arranged in 3×3 tables, with each cell representing one position on the webpage (Fig 8). Sixty-three combinations were obtained. The experimental results underwent statistical analysis to investigate the Kansei images of various combinations. Based on the literature and the car-related image vocabulary collected in this study, the three most representative image phrases were selected; these were sense of speed, stylishness, and steadfastness. Eventually, sense of speed was chosen as the image phrase to be tested in this study. Based on the common viewing angles and the literature, four representative viewing angles were selected (Figs 1, 2, 4 & 6). Images of three other viewing angles were then obtained through mirroring (Figs 3, 5 & 7). Each participant viewed 63 images on a computer screen. After viewing each image, he or she scored the image for its sense of speed on a 5-point Likert scale. This test aimed to determine the influences of different product viewing angles and product positions on a webpage on Kansei images. The participants were grouped by sex, dominant hand, and dominant eye to investigate the influences of their physical characteristics on Kansei images. A method of measuring dominant eye is commonly used. The first consists in placing both palms forward, and making a small hole by overlapping the first dorsal interossei of both hands and looking to a fixed point in the distance with both eyes through the hole and remaining in the state of being able to see the distant image while slowly drawing both hands toward the eyes; the small hole between the hands eventually approaches the dominant eye.

**Fig 1:** Car facing the front (VA1).

**Fig 2:** Car turned to the left (VA2).

**Fig 3:** Car turned to the right (VA3).

**Fig 4:** Car turned to the left rear (VA4).

**Fig 5:** Car turned to the right rear (VA5).

**Fig 6:** Car turned to the left front (VA6).

**Fig 7:** Car turned to the right front (VA7).

**Fig 8:** Positions of product images.

The research method of this study is stated as follows, including experimental samples, experimental independent variables, experimental dependent variables, and experimental control variables.

1. Experimental sample: The sample number is 50 people.
2. Experimental independent variables:
  1. Product perspective
    Representative photos from 7 perspectives (Figs 1–7)
  2. The position of the product on the web page
    Place the product photos in nine positions on the web page in a nine-grid manner (Fig 9).
    Therefore, there are 63 combinations of product perspectives and product positions on the web page.
3. Experiment dependent variable:
  1. Perceptual perception
    Perform the scoring of adjective vocabulary of each photo, and score on a five-point scale.
  2. Interview
    After the end of all the tests, the interviewees were counted on the criteria for the scoring of adjectives.
4. Experimental control variables:
  1. Configuration of space environment
    The subject can adjust the height of the chair and table to the most comfortable state, the computer is placed on the table for operation, and the lighting is sufficient.
  2. Screen configuration
    The screen picture is a gray scale car pattern, and the car positions are located at nine positions on the screen.
  3. Scoring of adjectives

**Fig 9:** Sense-of-speed scores assigned by all participants.

The task execution steps and procedures are unified, and the product photos are placed in nine positions on the web page in a nine-grid manner (Fig 9). Therefore, there are 63 combinations of product perspectives and product positions on the web page. Scoring the adjectives of 63 car designs.

In terms of experimental design, detailed explanations will be given on the preparation before the experiment, the steps of the experimental process, and the evaluation after the experiment.

1. Preparation before the experiment:
  Before the subject conducts the experiment, the researcher will first set up the equipment in the experimental environment and place the laptop on the desktop. In the environment tested by the subject, a quiet indoor environment with sufficient lighting and few interferences will be selected, and the subject shall be asked to adjust the height of their own seat and the most comfortable sitting posture on the table.
  On the laptop screen, the greater the difference between the graphics and the background color, the better the visual effect. The graphics of each car are grayscale, and the overall background is white.
  After the environment is set up, the description of the experiment is started. The researcher will explain the entire experiment in detail. After the explanation, the subject will be asked to ask questions. After the questioning is completed, let the subject take a short five-minute rest to ease Emotions, the part that starts the experiment.
2. During the experiment
  At each stage of the experiment, a round (a total of nine kinds) of scoring of adjectives will be scored. In the course of the experiment, the subjects recorded the confluence of adjective words in each screen.
3. After the experiment:
  When the subjects have completed the 7-stage experiment, they will be allowed to rest for five minutes. After the rest is over, they will be interviewed and recorded.

## Results

We applied a site research method and collected data through questionnaires. Convenience sampling was conducted in a university campus, and consent was obtained from all participants. In total, 50 university students aged between 18 and 24 years were recruited as participants. After retrieving the questionnaires, data processing and analysis were performed. The data were presented as descriptive statistics (i.e., means and standard deviations) and analyzed through an independent samples *t* test. The means reflected the difference between groups, and the standard deviations represented the estimated degree of dispersion among the participants. The independent samples t-test was used to examine whether speed perception differed significantly depending on physical characteristics (i.e., sex, dominant hand, and dominant eye). A *p* value of less than 0.05 was regarded as statistically significant.

The data obtained in this study underwent analysis and processing. Fig 9 presents the results of the sense-of-speed score for the 63 images with various viewing angles and positions. Fifty participants were recruited, and Table 1 shows their grouping results: 29 were men (58%) and 21 were women (42%); 45 were right-handed (90%) and 5 were left-handed (10%); 25 had the right eye as their dominant eye (50%) and 25 had the left eye as their dominant eye (50%). Six participants (12%) felt that the position of the car image on the webpage did not affect the car’s perceived sense of speed; three of these participants had the right eye as their dominant eye and three had the left. They all perceived the car in the images to be stationary. Eleven participants (22%) felt that the position of the car image on the webpage almost did not affect the car’s perceived sense of speed; eight of these participants had the left eye as their dominant eye (32% of all participants with the left eye as the dominant eye) and the remaining three had the right eye as their dominant eye (12% of all participants with the right eye as the dominant eye). These participants gave approximate scores (± 1 point) for sense of speed in car images with the same viewing angle but different positions. The remaining 39 participants (78%) considered that the car’s viewing angle and the position of the car image on the webpage both affected the car’s perceived sense of speed.

**Table 1:** Distribution of sample groups.

Sex		Dominant hand		Dominant eye	
**Men**	Women	Right-handed	Left-handed	Right-eye-dominant	Left-eye-dominant
**29**	21	45	5	25	25

Figs 9–15 show the sense-of-speed scores that the various participant groups assigned to car images. The sense-of-speed scores ranged from 1 to 4 points and were divided into six intervals of 0.5 points. Each score interval is represented by a color shade; darker color indicates a stronger sense of speed.

**Fig 10:** Sense-of-speed scores assigned by men.

**Fig 11:** Sense-of-speed scores assigned by women.

**Fig 12:** Sense-of-speed scores assigned by right-handed.

**Fig 13:** Sense-of-speed scores assigned by left-handed.

**Fig 14:** Sense-of-speed scores assigned by right-eye-dominant.

**Fig 15:** Sense-of-speed scores assigned by left-eye-dominant.

When all participants had been considered (Fig 9), the highest sense-of-speed score for each viewing angle was obtained as follows: 1.88 points for viewing angle (“VA” hereafter when referring to specific angles) 1 and position (“P” hereafter when referring to specific positions) 5; 2.18 points for VA2, P4; 2.22 points for VA3, P6; 2.94 points for VA4, P1; 2.94 points for VA5, P3; 2.36 points for VA6, P7; and 2.56 points for VA7, P9. Of all 63 images, the highest sense-of-speed score—2.94 points—was observed for the combinations of VA4, P1 and VA5, P3, whereas the lowest score—1.48 points—was observed for the combination of VA1, P1. The results revealed that perceived sense of speed was derived from the distance between the front of the car and the screen boundary. That is, the closer the car front is to the screen boundary, the faster the viewer perceives the car to be, and thus a stronger sense of speed is generated.

When the participants were grouped by sex, the men assigned their highest sense-of-speed score (3.03 points) at VA4, P1 and their lowest at VA1, P7 (1.38 points) (Fig 10). The women assigned their highest sense-of-speed score (3.05 points) at VA4, P4 and VA5, P3 and their lowest at VA1, P2 (1.48 points) (Fig 11). The minimum score variance among the men was determined at VA3, indicating that the men exhibited their highest consistency at this angle; by contrast, the women exhibited their highest consistency at VA1 (Table 2).

**Table 2:** Means and variance of sense-of-speed scores.

sample group viewing angle	All (*n* = 50)	Men (*n* = 29)	Women (*n* = 21)	Right- handed (*n* = 45)	Left- handed (*n* = 5)	Right-eye- Dominant (*n* = 25)	Left-eye- dominant (*n* = 25)
VA1	1.63 (Mean)/ 1.19 (variance)	1.53/1.23	1.77/1.09	1.59/1.19	1.98/1.02	1.57/0.94	1.69/1.43
VA2	1.95/1.22	1.66/0.81	2.34/1.51	1.93/1.22	2.16/1.13	1.96/1.09	1.94/1.35
VA3	2.04/1.18	1.84/0.79	2.32/1.59	2.01/1.22	2.27/0.79	1.99/1.08	2.09/1.28
VA4	2.58/1.82	2.45/1.81	2.75/1.79	2.54/1.85	2.89/1.51	2.37/1.66	2.79/1.90
VA5	2.62/1.87	2.48/2.00	2.81/1.63	2.59/1.89	2.84/1.63	2.33/1.50	2.90/2.08
VA6	2.18/1.63	2.15/1.74	2.23/1.47	2.05/1.48	3.31/1.54	2.08/1.29	2.28/1.95
VA7	2.40/1.56	2.31/1.75	2.53/1.28	2.32/1.42	3.20/2.12	2.15/1.30	2.66/1.70

When the participants were grouped by their dominant hands, the right-handed group assigned their highest sense-of-speed score (2.96 points) at VA4, P1 and VA5, P3 and their lowest at VA1, P4 (1.47 points) (Fig 12). The left-handed group assigned their highest sense-of-speed score (3.80 points) at VA6, P5; VA6, P7; and VA7, P7 and their lowest at VA1, P1 (1.40 points) (Fig 13). The right-handed group showed their highest consistency for sense of speed at VA1, whereas the left-handed group were most consistent at VA3 (Table 3). The statistical results suggested that the dominant hand affected the sense of speed derived from the direction of the car.

**Table 3:** Regression result for the VA2, P3 combination.

**Regression statistics**	
R	0.40293
R2	0.16235
Adjusted R^2^	0.14490
SE	1.00327
n	50

**ANOVA**	df	SS	MS	F	P
Regression	1	9.36472	9.36472	9.30362	0.00371
Residual	48	48.3152	1.00656		
Total	49	57.68			
	Coefficient	SE	t	P
Intercept	2.4285	0.21893	11.09274	7.62E-15
Xs	-0.8768	0.28747	-3.05018	0.003717

When the participants were grouped by their dominant eyes, the right-eye-dominant group assigned their highest sense-of-speed score (2.88 points) at VA4, P1 and their lowest at VA1, P2 (1.36 points) (Fig 14). The left-eye-dominant group assigned their highest score (3.12 points) at VA5, P3 and their lowest at VA1, P1 (1.40 points) (Fig 15). The right-eye-dominant group was most consistent for sense of speed at VA1, whereas the left-eye-dominant group was most consistent at VA3 (Table 2).

Regarding pairs of viewing angles obtained through mirroring, all participants perceived different speed levels for the two angles in each pair. Specifically, based on the participants’ average sense-of-speed scores, VA2 < VA3, VA4 < VA5, and VA6 < VA7; the sense of speed generated when the car was facing right was greater than that generated when the car was facing left (Fig 9). A comparison of the men’s average sense-of-speed scores for mirrored angle pairs revealed that VA2 < VA3, VA4 < VA5, and VA6 < VA7; the sense of speed generated when the car was facing right was greater than that generated when the car was facing left (Fig 10). A comparison of the women’s average sense-of-speed scores for mirrored angle pairs revealed that VA2 ≈ VA3, VA4 < VA5, and VA6 < VA7; the sense of speed generated when the car was facing right was greater than that generated when the car was facing left (Fig 11). A comparison of the right-handed group’s average sense-of-speed scores for mirrored angle pairs revealed that VA2 < VA3, VA4 < VA5, and VA6 < VA7; the sense of speed generated when the car was facing right was greater than that generated when the car was facing left (Fig 12). A comparison of the left-handed group’s average sense-of-speed scores for mirrored angle pairs revealed that VA2 < VA3, VA4 > VA5, and VA6 > VA7 (Fig 13). A comparison of the average sense-of-speed scores of the right-eye-dominant group for mirrored angle pairs revealed that VA2 ≈ VA3, VA4 ≈ VA5, and VA6 < VA7 (Fig 14). A comparison of the average sense-of-speed scores of the left-eye-dominant group for mirrored angle pairs revealed that VA2 < VA3, VA4 < VA5, and VA6 < VA7; the sense of speed generated when the car was facing right was greater than that generated when the car was facing left (Fig 15).

In terms of sex, the speeds perceived by women for all seven viewing angles were higher than those perceived by men. Regarding the dominant hand, the left-handed group perceived higher speeds for all seven viewing angles than did the right-handed group. Regarding the dominant eye, the left-eye-dominant group perceived higher speeds for all seven viewing angles than did the right-eye-dominant group (Table 2).

A multiple regression analysis was conducted with speed perception (determined using Kansei evaluation) as the dependent variable and physical characteristics (sex, dominant hand, and dominant eye) as the independent variables. The results showed that just one of physical characteristics is significant for speed perception. A simple linear regression analysis was then performed with speed perception as the dependent variable and one of the physical characteristics as the independent variable.

The simple linear regression analysis was used to construct a regression equation between speed perception and physical characteristics (sex, dominant hand, and dominant eye). When sex was the independent variable and speed perception was the dependent variable, the regression equation exhibited satisfactory explanatory power for speed perception with the following combinations of experimental conditions: VA2, P3; VA2, P4; VA2, P5; VA2, P6; VA2, P8; VA2, P9; VA3, P3; VA3, P8; and VA3, P9. When dominant hand was the independent variable and speed perception the dependent variable, the regression equation showed satisfactory explanatory power for speed perception with the following combinations of experimental conditions: VA6, P5; VA6, P6; VA6, P7; VA6, P8; VA6, P9; and VA7, P7. When dominant eye was the independent variable and speed perception the dependent variable, the regression equation demonstrated adequate explanatory power for speed perception with the following combinations of experimental conditions: VA4, P5; VA5, P9; and VA7, P2.

For example, the regression result for the VA2, P3 combination was shown in Table 3, and the regression equation was as follows:

$$Y_{VA2P3}=2.4285-0.8768Xs$$

For men, Xs = 1; for women, Xs = 0.

This study conducted interviews to determine the factors that affected the participants’ perceived sense of speed. In addition to intuition, other factors are detailed as follows:

1. The sense of speed for the front view (VA1) originated from the sense of the car coming toward the viewer. Cars positioned in the top row (P1–P3) and bottom row (P7–P9) of the webpage created different senses of speed among the participants, namely that the cars in the top row appeared relatively far away, whereas those in the bottom row appeared relatively close; therefore, the top row produced a relatively slow sense of speed, whereas the bottom row produced a relatively fast sense of speed. However, some participants considered that the middle row (P2, P5, & P8) produced the greatest sense of tension, thereby creating a fast sense of speed. Some participants even posited that the middle column (P4–P6) posed the greatest sense of tension, and thus produced a fast sense of speed; in addition, some perceived the greatest sense of tension in the middle cell (P5), and thus considered this position to entail the fastest sense of speed.
2. Sense of speed may have been produced for the front view because of the streamlined car front design.
3. Sense of speed for the side views (VA2 and VA3) was derived from the distance between the moving direction of the car and the screen boundary. When the front of the car was close to the screen boundary, the viewer would likely feel that the car was about to drive out of the screen, and thus perceive a fast sense of speed.
4. Regarding the factors that influenced sense of speed for 45° views, some participants considered that these factors were identical to those that influenced the sense of speed for the side views; some participants felt that each car whose moving direction is parallel to the diagonal produced a relatively fast sense of speed (e.g., when the car was facing the left rear, the sense-of-speed scores were P1 > P5 > P9 > other positions). Some participants considered that the distance between a car’s projection point on the diagonal and the screen boundary affected said car’s perceived sense of speed (e.g., when the car was facing the left rear, the sense-of-speed scores were P1 > P2 and P4 > P3, P5, and P7 > P6 and P8 > P9). Nevertheless, some participants held the opposite point of view—they considered that cars in 45° views appeared bulky because their front or rear was enlarged in the perspective, which produced a relatively slow sense of speed.
5. The middle cell (P5) obtained a relatively satisfactory sense of speed for all viewing angles.

## Discussion

This study mainly focused on determining the influences of various product viewing angles and webpage positions on consumers’ Kansei images. Representative viewing angles and Kansei phrases were identified through a literature review. A selected representative Kansei phrase, namely sense of speed, was then combined with various viewing angles and positions to test the participants’ Kansei images by conducting a questionnaire. Taking car appearance as an example, the highest sense-of-speed score was observed for the combinations of VA4, P1 and VA5, P3. Regarding car images with different viewing angles, the fastest sense of speed was observed in various webpage positions. Both the moving directions suggested by various viewing angles and being situated on the edge of the webpage contributed to enhancing the sense of speed. The results of this study could serve as a reference for webpage design staff in determining viewing angles and positions for product display. This study proposed methods for analyzing the influences of product presentation angles and webpage positions on consumers’ Kansei images, and investigated the influences of consumers’ physical characteristics on their Kansei images. The results revealed that the participants’ physical characteristics did affect their Kansei images. This method could also apply to research on other products focusing on other Kansei phrases. The following findings were derived from the statistical analysis of the data obtained in this study:

1. When all the participants had been considered, the score distribution results regarding the highest sense of speed for various viewing angles revealed that the closer a car was to the screen boundary, the stronger the sense of speed became. In addition, the sense of speed generated when the car was facing right was stronger than that generated when the car was facing left.
2. Of the participants who considered that the position of the car image on the webpage barely affected the car’s sense of speed, the left-eye-dominant group outnumbered the right-eye-dominant group.
3. Sex, dominant hand, and dominant eye all affected the participants’ perceptions of a car’s sense of speed.
4. The results of the analysis of variance indicated that individual differences in the right-eye-dominant group were more minor than those in the left-eye-dominant group, and individual differences among the participants related to the car’s sense of speed for the front and side views were more minor than those for the 45° views.
5. The results revealed that consumers’ physical characteristics do affect their Kansei images for products. Conventional marketing platforms cannot adjust their content for different customers; however, online marketing platforms can document customers’ physical characteristics to provide them with personalized product displays in order to cater to their Kansei image preferences. These research findings could be applied to online shopping platforms, which could attract more diverse groups of clients by adjusting product display angles and product positions on webpages based on consumers’ physical characteristics and preferences.

## Conclusions

Previous studies on Kansei engineering have not explored the influence of consumers’ dominant hands and eyes on their Kansei images. In this study, the influence of product viewing angle and position (on a webpage) on consumers’ Kansei images was determined; the influence of consumers’ physical characteristics (sex, dominant hand, and dominant eye) on their Kansei images was also explored. The following conclusions were drawn: (1) viewing angle, (2) the position of the product on the webpage, and (3) some participant physical characteristics affected the participants’ Kansei images. In summary, online marketing platforms can record shoppers’ physical characteristics to provide them with personalized product displays and cater to their Kansei image preferences.

These research findings can be applied in online shopping platforms by adjusting product display angles and product positions on webpages according to consumers’ physical characteristics and preferences, which could attract more diverse groups of clients.

Because the sample groups had different characteristics, the statistical results of different sample groups may be different. However, this method was still applicable. Future studies should select different target groups for sampling, questionnaire surveys, and statistical analyses or use different products and adjective words for research.

## Supporting information

S1 Table Sense-of-speed scores. (XLS)
